# Analysis of the Path and Relationship between Movement-Style Environmental Governance and Political Potential Energy Integration and Isomorphic Transformation

**DOI:** 10.1155/2022/1555102

**Published:** 2022-09-30

**Authors:** Yinglian Sun

**Affiliations:** School of Marxism, Research Institute for the Development of Socialism with Chinese Characteristics, Southeast University, Nanjing 210018, China

## Abstract

As a theoretical research framework for analyzing the governance of China, political potential energy is a concept with local discourse characteristics. Political potential energy highlights the comprehensive leadership ability of the Chinese Communist Party in the ruling process. It has profound political and dynamic connotations, and it is reflected in all aspects of the Chinese Communist Party's governance. The linkage logic between movement-style environmental governance and political potential energy suggests that the gathering of political potential energy and scientific placement are crucial. Political potential energy needs to be supported by certain rules and systems, and local autonomy must be fully respected. Therefore, by exploring the relationship between movement-style governance and political potential energy and the path of homogeneous transformation, these issues are worth exploring, which are related to the major theme of national governance capacity and governance system modernization.

## 1. Introduction

“No major change in a century” is a comprehensive response to the uncertainty and turbulence of current international development. The world trend, value, and order are continuously cultivated and formed in the process of change. The influence of the rule of China has been continuously highlighted, linking the “broken” and “established” sides of the strait of great changes. Chinese wisdom shows its own charm in the reality of the “broken” and “established” cross-strait structures [1]. From the perspective of environmental governance in China's overall strategy, the development of the western region plays a very significant strategic position in the long-term development of China's social and economic development. Environmental protection and construction has become the fundamental task of western development. Comprehensive measures should be taken to “return farmland to forests, close mountains for greening, use grain for relief, and individual contracting [2].”

Political potential energy“ is the institutional resource accumulated by the Communist Party of China in the long-term revolution and construction process. Political potential energy refers to the development trend and influence energy of a political organization or group itself and presented in its political life and political movement. “Movement warfare” is the key to the transformation of political potential energy into governance effectiveness [3].

This paper mainly analyzes the relationship between movement governance and political potential, finds out the trend of movement environmental governance and political potential of the movement, and analyzes the media and the problems in the process of environmental governance, which has important guiding significance for promoting national environmental governance.

## 2. State of the Art

### 2.1. Movement Governance

The research on movement-style governance has been going on, and many scholars have explored this topic from multiple perspectives and methods. In 2004, the research subject heading of domestic movement-style governance first appeared in the public literature [4]. Based on the rectification analysis of the Beijing Office, Hongguang believes that since the reform and opening, it has undergone the rectification of the Beijing Office in the form of movement-style governance many times, and practice has shown that sports-style governance has become a regularized government governance method, showing the cyclical characteristics of stylization and irregularity. After 2007, more scholars entered into the study of movement-style governance, especially in recent years, movement-style governance coincides with the research theme of national governance system and governance capacity and has become an important incision for analyzing governance form, governance capacity, and governance modernization. The current academic research on movement-style governance continues to deepen, not only focusing on expounding the concept and causes of movement-style governance, but also in the process of researching the effect of movement-style governance. It can be said that a fundamental turn has taken place as a whole [5].

### 2.2. Political Potential

Political potential is one of the important factors to promote the implementation of the system and the implementation of public policies. As one of the manifestations of the political elements of China's governance, political potential energy affects the ability of environmental public policy to monetize. The most important manifestation is that it has an impact on the willingness of actors to implement public policies through the hierarchical structure and top-down power operation [6]. Political potential, a research framework for analyzing China's governance, has obvious characteristics of local discourse. The first scholar to put forward political potential energy was Kong Fanbin. Although political potential is a new concept in the theoretical circle, it can better explain the Chinese governance experience and Chinese characteristics of public policy implementation [7]. Third, the political potential fully demonstrates the multiattribute governance and hierarchical governance issues derived from the long-term implementation of public policies in China. The political distance can bring a “Curse” to the executive agency, which can break through the previous bureaucratic division and inertia, thereby enhancing the executive power and ensuring the realization of policies as soon as possible.

As shown in Figure 1, political potential energy mainly includes four dimensions: value political potential energy, institutional political potential energy, structural political potential energy, and unified political potential energy [8]. In the process of comprehensive environmental governance in China, the transformation relationship between political potential energy and governance effectiveness is shown in Figure 2. By giving full play to the advantages of political potential energy in four dimensions and using the political potential energy of local party committees and governments, the campaign-style environmental governance is promoted effectiveness [9].

### 2.3. Movement Governance and Political Potential

The assistance of cases can fully demonstrate the role of political potential energy. Political potential energy has a comprehensive effect on the implementation of public policies, local governance, and governance of attributes (environmental pollution, health protection, law enforcement, etc.) [10]. Sport-style governance has gradually become an important analytical paradigm for social governance practice in social transformation, and the institutional environment and practice mechanism of movement-style governance in the reconstruction of China's order in transition are embodied in the hierarchical coordination mechanism under the pressure-based system, the political mobilization mechanism under the championship system, and the administrative absorption mechanism under the bureaucratic system at the section level. In the movement-style governance, in recent years, it has mainly focused on environmental law enforcement, environmental inspections, environmental pollution, and environmental policy implementation. Therefore, it is of certain significance and value to analyze the linkage logic between movement-style environmental governance and political potential energy with the aid of relevant cases of environmental governance.

## 3. Analysis of the Relationship between Movement-Style Governance and Political Potential Energy

### 3.1. Integration: The Logical Starting Point of the Relationship between Movement-Style Environmental Governance and Political Potential

The one-way study on the governance of sports style and political potential energy makes the relationship between them fuzzy. Because the concept of political potential energy has only appeared in recent years, political factors cannot exceed the threshold in sports governance, which has been regarded as sports governance. The fuzziness of political factors and sports style governance are interrelated, leading to many studies unable to explain sports style governance in a more in-depth and innovative way from the perspective of political factors, making it difficult for many studies to deeply analyze and innovate sports style governance based on the political level [11]. Therefore, in the governance of sports environment, we can make a more systematic and image observation on the change and appearance of political potential energy. The effectiveness of nontraditional governance is the key function of sports environmental governance. Compared with conventional governance, the key characteristics of sports governance are the allocation of resources, integration, and diversification of governance means [12].  Figure 3 shows the early warning and coordination mechanism and process of the water quality detection system in the process of governance of a certain water area.

The motive force of the campaign type environmental governance lies in surmounting the old relationship of division, breaking bureaucracy, mobilizing various resources, and quickly realizing the governance efficiency. It is the core of political potential energy to determine the political attribute in the implementation of policies. There is no big difference between the political elements and the political potential energy. There are also low and high political potential energies. If there is a higher political potential energy, there will be a larger policy potential energy, and it may have a better ability to realize the policy. The political potential will have an impact on various themes and elements of the campaign style environmental governance, such as bureaucratic cooperation, official attitude, and resources [13]. In fact, we can regard formal energy as a unique invisible color of public policy.  Figure 4 shows the organizational structure relationship of the comprehensive management work headquarters of an administrative region in the Xin'an River management action [14]. It can be seen that the government plays an extremely important role in the water environment management of the river basin, and different levels of government have different political potentials.

### 3.2. Transformation Trend: Movement-Style Environmental Governance and Changes in Political Potential Energy

#### 3.2.1. Mutual Promotion: Movement-Style Environmental Governance and the Trend of Political Potential

The dynamic environmental governance interacts with political potential energy. There is a close relationship between political potential energy and movement type environmental governance. Environmental governance tends to be standardized due to political potential energy. Especially when the potential energy is accumulated to a corresponding level, it can be quickly released in a short time. Governance is generally squeezed into the motion trajectory [15]. When governance moves to a movement-style environmental governance model, although it may cause a series of consequences, the governance efficiency is low, and the administrative cost and resource consumption are not proportional to the final sense of governance gain, but the movement-style environmental governance gives the government a wealth of learning experience. Process learning is always going on [16]. As an active subject, the government obviously understands that every use of campaign-style governance will lead to the consumption of some organizational resources of the political party. If the campaign-style governance is not effective, it will even lead to some authoritative resources. Moreover, once the movement-style governance is included in the daily scope, it will increase the operating cost of the organization and increase the people's expectations for the government. The large gap between expectations and reality often weakens the people's trust in the party and the government. Therefore, after the combination of political potential energy and movement-style environmental governance, whether the final trend is to enter into the category of movement-style governance or into the conventional governance system, the connection between the two will become clearer. The movement “governance mode can solve the problem of the central government's power out of control over the grass-roots government, standardize the” flexible use “ of the grassroots government to the central government policy, and become an important tool to coordinate the relationship between the central government and the grass-roots government. How to use the political potential energy to better serve the Modernizing the governance system and governance capacity, avoiding the movement of governance, continuing to consolidate and develop the advantages of the socialist system with Chinese characteristics, and manifesting the “rule of China“ with “China's system” are new issues that need to be faced in the future.

#### 3.2.2. The Joint Transformation and Enlightenment of Movement-Style Environmental Governance and Political Potential

The Xin'anjiang governance model has been incorporated into the conventional governance system with the development of time. The distribution is gradually balanced. For example, Anhui Province has upgraded the governance of Xin'an River to the “No. 1 Project” of an ecologically strong province, the establishment of leading groups from the provincial to the municipal level, the evaluation indicators are inclined to the ecology (as shown in Table 1), and more than 70 policy documents have been issued. Various local initiatives reveal the gradual dispersal of political potential energy in the local area and evolve into a lasting driving force for the conventional governance of the Xin'an River [17].

## 4. Case and Empirical Analysis

Sport-style governance is naturally linked to political factors, and movement-style governance in environmental governance is often displayed in front of people, such as various “shutdown actions” and “special actions” in news reports, and “100-day battles” for environmental protection governance initiated or launched in many places, aiming at the actual situation of the integration process of movement-style environmental governance and political potential energy. The author analyzes the case of movement-style governance in Taihu Lake area of Jiangsu province and reveals various political elements and political potential energy through environmental governance in Taihu Lake area.

### 4.1. Movement-Style Environmental Governance and Political Potential Energy Integration Process

Taihu Lake has more than 2300 square kilometers of water area and 37,000 square kilometers of watershed area, which is the third largest freshwater lake in China. From 1991 to 2004, the first stage of harnessing Taihu Lake invested more than 10 billion yuan [18]. On December 31, 1998, the provincial and municipal governments of Jiangsu, Zhejiang, and Shanghai reported the final completion and inspection results of the “zero point action” governance work successively. Prior to New Year's Day in 1999, the official announced that governance had “basically achieved its phased goals” [19]. However, in 2001 and 2003, researchers Zhang and Sun analyzed the changes of water quality before and after the “Taihu Zero Action”. The results are consistent and do not improve pollution effectively. Under such sports-style environmental governance, all kinds of political potentials and factors quietly integrate. First, a pressure transfer conference was held. The Environmental Protection Committee of the State Council held a meeting on environmental law enforcement inspection in April 1996, which was attended by ministries of the State and leaders of the three provinces and cities of Jiangsu, Zhejiang, and Shanghai. This can be regarded as an early accumulation of pressure and, in fact, a wind guide for political mobilization. Another is the clamor of publicity and red header documents. This action originated from the “Ninth Five-Year Plan” and the plan for prevention and control of water pollution in Taihu Lake in 2010. After that, the State and Jiangsu Province successively promulgated the regulations on water pollution. The Taihu Zero Achievement Action became a national focus in 1999, attracting more than 30 news organizations. CCTV alone dispatched 33 people and more than 100 journalists. Red hair documents and public opinion have fully mobilized and activated various sleep resources. Thirdly, the Coordinating Leading Group should be set up. Leading groups include coordination and leadership groups at different levels as well as committee working groups. The division of work among the leading groups is shown in Table 2.

In the “Focus on Taihu Lake Zero-point Compliance” campaign, the State Environmental Protection Administration established the “Focus on Taihu Lake” front-line headquarters to command the “Zero-point compliance” action. Finally, political incentives and promotions and the championship system also play an important role in sports-style environmental governance. Sports-style environmental governance is performance-oriented and the central government sets goals and rules, top-down political incentives, and local government officials. The promotion game interacts with each other. The championship system is inherently compatible with the political movement methods of the general society. The Taihu Zero Action Command Center is divided into two groups to conduct inspections. During the zero-point action, personnel from the party, government, and environmental protection departments in Jiangsu, Zhejiang, and Shanghai go to the scene. There is a whole set of potential political expressions of promotion, incentive, and punishment behind the inspections, such as inspecting the enterprises that meet the emission standards. The specific division of labor of the member systems of each headquarters in the region is shown in Table 3. It is in this process that the administrative departments are responsible for their respective responsibilities, efficiently complete the various intelligences assigned by the superiors, and ensuring the completion of the central goals as scheduled.

Therefore, in the process of movement-style environmental governance, the integration process of various political elements and political potential energy is also the three advanced processes of the role of political potential energy [20]: the first stage, “the party's leadership is present”; the second stage, “building power”; the third stage, “taking advantage of the situation to make things happen”. In the context of social transformation, the dilemma of movement-style governance is embodied in the dilemma of “movement-style” governance and the practice of “bureaucratic system”, the dilemma of “policy adaptation” and “conspiracy behavior” in movement-style governance actions, and the dilemma of “governance theaterization” and “theater politics” based on the orientation of “governance performance” in movement-style governance. The Chinese empirical logic of China's grassroots social governance changes and its modern transformation reflects the dual-track coordination from movement-style governance to normal governance, movement-style governance to section-level operation, participatory governance under the cogovernance of multiple subjects, and the shift of grassroots network governance in the interactive field of actors. Through the accumulation of political potential energy in three stages, it plays a role in deterring, preventing, or changing the direction of travel for “contrarians”, it plays a role in promoting and motivating “followers”, and driving the continuous movement of environmental governance to in-depth development. “Taihu Lake Zero Action” as a movement-style environmental governance, the pressure transmission of the meeting can be classified as the first stage of political potential energy “party leaders are present”, including the leaders of national ministries and commissions and the leaders of Jiangsu, Zhejiang, and Shanghai during the meeting. The red-headed document and the establishment of a leadership coordination group belong to the second stage of political potential energy “building power”, which aims to unify ideas, release signals, and divide and integrate governance tasks and build the third stage of political potential energy “taking advantage of the situation to make things happen” base.

### 4.2. Movement-Style Environmental Governance and the Media of Political Potential

Isomorphism refers to a certain degree of similarity between things in structural composition or structural properties, so that the change and development of things are affected by common causes, so that things can integrate and promote each other, rather than mutually exclusive, that is, the media of movement-style environmental governance and political potential. In the case study, the ecological compensation sample of the Xin'an River basin is selected, the trace and analysis process of the case can help to more comprehensively explore the similarity between the movement-type environmental governance and the political potential energy medium, and further prospect the future development and change of the sports-based environmental governance. The Xin'an River originates from Huangshan Mountain in Anhui province, and the average outbound water volume accounts for more than 68% of the inflow water of the downstream Qiandao Lake in Zhejiang province. The water quality of the Xin'an River Basin is related to the ecological security of the entire Yangtze River Delta. At the beginning of the 21st century, with the accelerated development of Huangshan's industrialization and urbanization, a large amount of sewage and garbage flowed into Qiandao Lake through the Xin'an River, and the ecological security of the basin faced severe challenges. As early as 2006 and 2007, the Ministry of Finance and the former Ministry of Environmental Protection organized the two provinces of Anhui and Zhejiang to conduct in-depth investigations on the ecological problems of the Xin'an River basin. Both provinces attached great importance to the issue of ecological compensation in the Xin'an River Basin, but each has his own opinion. In February 2011, Comrade Xi Jinping, then a member of the Standing Committee of the Political Bureau of the CPC Central Committee and vice-president of the state, made important instructions, emphasizing that “Qiandao Lake is an extremely rare high-quality water resource in my country, and it is of great significance to strengthen the protection of Qiandao Lake's water resources. Repeating the mistakes of pollution first and then treatment,” and hoped that “Zhejiang and Anhui provinces should focus on the overall situation, control pollution from the source, and take the road of mutual benefit and win-win”. In September 2011, the “Xin'an River Basin Water Environment Compensation Pilot Implementation Plan”, which was researched and formulated by the Ministry of Finance and the Ministry of Environmental Protection in conjunction with Anhui and Zhejiang provinces for more than two years, was officially issued. After the two rounds of pilot projects, the water quality in the upper reaches of the Xin'an River from 2012 to 2017 was generally excellent, the water quality of Qiandao Lake remained stable in the second category, and the trend of water quality deterioration was reversed. The mechanism is gradually normalized.

In the Xin'an River governance model, there is a background of movement-style environmental governance. Before the governance, the water quality of the basin was poor and the governance was difficult. It involved the coordination of Anhui and Zhejiang provinces. Only by strengthening the political power of the central government could ecological compensation in the basin be achieved. Among them, the instructions of the important leaders of the central government played a decisive role, and the Xin'anjiang governance model was fully developed after the instructions of Comrade Xi Jinping, then member of the Standing Committee of the Political Bureau of the Central Committee and vice-chairman of the state. In terms of the assessment reward and punishment mechanism, the assessment indicators for Huangshan focus on ecological protection. In the performance assessment system of relevant township departments in Chun'an County, ecological indicators account for about 70%. The Xin'an River governance model is different from the “zero-point action” of Taihu Lake governance. The Xin'an River governance model has been gradually normalized after two rounds of pilots, while the “zero-point action” of Taihu Lake governance has evolved into a typical movement-based environmental governance. The development trend of the government is different, but political potential has played an important role in it. In the Xin'anjiang governance model and the Taihu Lake governance “Zero Action”, the media of political potential is different. After filling the gap, the presence of leaders, the superposition of documents, the incentive mechanisms, media clamor, etc. are not only the media of political potential energy, but also an important measure of movement-style environmental governance or a key link in the governance process [5]. The formation process and key links of movement-style environmental governance are infused with the media of political potential energy and can be roughly classified into three development stages of political potential energy, and the three development stages of political potential energy are also movement-style environments. The process of formation, development, and change of governance as an open field, it will not rule out more isomorphic media entering the field in the future, which will continue to influence the process of movement-style environmental governance and the development of political potential as shown in Figure 5.

## 5. Conclusion

Under the background of the unprecedented strengthening of the central environmental protection authoritarianism, campaign-based governance characterized by breaking conventions, resource mobilization, and special actions is becoming the norm of local environmental work and is beginning to be normalized. By analyzing the relationship between movement-style governance and political potential, this paper identifies the trend of movement-style environmental governance and political potential promoting each other.

The interaction between movement-style environmental governance and political potential energy expands the existence space of political potential energy. Movement-style environmental governance is still being staged in China from time to time, but large-scale movement-style environmental governance, especially the rapid accumulation and release of high-level political energy from the central government, is no longer common. The local operation of political power is gradually normalized. In the process of remobilization of microregional movement-style environmental governance, the local potential energy layer is constantly acting, thus contributing to the remobilization. The reason is that when the local political potential is weakened, the “movement-style” means dissolves into daily administration, and its governance performance gradually declines. “Ratchet effect”, the governance process is caught in “involution”.

## Figures and Tables

**Figure 1:** Dimensions of political potential.

**Figure 2:** The transformation framework of political potential energy and environmental governance effectiveness.

**Figure 3:** Early warning and coordination process of water quality detection system in a water area governance action.

**Figure 4:** Organizational relationship of the comprehensive management work headquarters in a district.

**Figure 5:** Isomorphism of movement-style environmental governance and political potential media.

**Table 1:** Annual performance evaluation index system and scoring table of government departments (parts).

Target type	First-level indicator	Secondary indicators	Three-level indicator	Score	Target requirements and specific indicators	Responsible unit
Functional goals	5. Ecological construction	(13) Pollution control	38. Water resource management	12	The annual average water quality of each section in the watershed in area A will get full marks, otherwise, it will be scored according to the monitoring frequency of meeting the standard, that is: actual score = assigned score^∗^ (frequency of meeting the standard/total monitoring frequency). [assessment of each town (street)]	District environmental protection bureau
			40. Special treatment of N River	15	(1) Submit materials on time (2 points), (2) identify and verify the pollution prevention situation and delineate the no-holding area (3 points), (3) ecological farming (1.5 points), (4) comprehensive utilization rate of manure (2 points), (5) normal operation of the sewage treatment plant (3 points), (6) add phosphorus removal process to sewage treatment facilities (2 points), (7) construction of automatic water quality station (1.5 points)	

**Table 2:** Division of responsibilities of the working group (part).

Water-wading enterprises, small scattered pollution enterprises governance working group	Strengthen the special governance of water-related polluting enterprises and small scattered polluting enterprises, conduct a comprehensive investigation of water-related polluting enterprises, and resolutely ban illegally operating water-related enterprises.
Aquaculture pollution control working group	Accelerate the demolition of livestock farms (households) in prohibited areas of the river basin; speed up the construction of harmless treatment facilities for livestock and poultry; investigate and ban illegal animal slaughtering points.

Rural domestic sewage treatment working group	Effectively speed up and improve the construction of the supporting pipe network for sewage treatment facilities; complete the interception of all the direct discharge outlets of domestic sewage in the built-up area; strengthen the management and control of phosphorus in living sources.

**Table 3:** Division of responsibilities of member system (part).

District environmental protection bureau	Responsible for coordinating and promoting the comprehensive management of the water environment in the basin, strengthening the environmental supervision of industrial enterprises, livestock, and poultry breeding pollution control facilities and the operation of urban sewage and domestic waste treatment facilities, and improving the construction of water quality and environmental monitoring sites in the basin and monitoring and early warning work. Responsible for the daily work of the joint meeting.
District development and reform bureau	Responsible for guiding relevant investments at the same level, promoting market-based financing, increasing policy and project support for comprehensive water environment management in the basin, and guiding the green development of the basin.

District finance bureau	Responsible for coordinating relevant funds to increase investment in the comprehensive management of the water environment in the basin, and strengthen the supervision and management of the use of funds.

District aquatic animal husbandry and veterinary bureau	Responsible for guiding and promoting the transformation of ecological breeding models and comprehensive utilization of breeding waste, strictly controlling the scale of pig breeding in the basin, organizing the implementation of standardized construction of large-scale breeding enterprises, and guiding the comprehensive utilization of breeding pollutants in the agricultural field.

Territory town street	Specifically responsible for the implementation of comprehensive management measures and project construction.

## Data Availability

The labeled data set used to support the findings of this study is available from the corresponding author upon request.
